# Formation Mechanism of Microbial Diversity in Artificial Intelligence Devices due to Intermediate Disturbance by Low-Dose UV Radiation for Complementary Medicine

**DOI:** 10.1155/2022/2874835

**Published:** 2022-09-09

**Authors:** Junjie Ye, Yang Yang, Juanyi Wang, Jingyu Han, Lihong Zhang, Tianrun Gong, Yi Zhang, Xiaodong Xing, Chen Dong

**Affiliations:** ^1^Department of Health Service and Management, School of Sport Management, Shandong Sport University, Jinan 250102, China; ^2^School of Graduate Education, Shandong Sport University, Jinan 250102, China; ^3^Shandong Provincial Hospital, Jinan 250021, China; ^4^Shandong Maternal and Child Health Hospital, Jinan 250014, China

## Abstract

The development of artificial intelligence devices in the complementary medicine field is rapid and the surface microbial diversity pollution was found with periodic low-dose ultraviolet radiation (LDUVR). Since artificial intelligence devices do not have enough different types of substrates for microbial communities, it is unclear how the great microbial diversity can emerge and persist, as this clearly defies the competitive exclusion principle of ecology. In this study, the 5 most common genera in the artificial intelligence devices, *Escherichia*, *Pseudomonas*, *Streptococcus*, *Staphylococcus* and *Aeromonas* have been sampled without and with periodic LDUVR, respectively. A new hypothesis was put up to clarify the construction and maintenance process of high microbiological diversity in artificial intelligence devices by comparing and evaluating the variations between the dynamic response characteristics of their relative abundances in the two scenarios as follows: the periodic LDUVR can be regarded as an adverse factor with intermediate disturbance, causing stronger microbial stochastic growth responses (SGR) which would inevitably give rise to stronger random variation of the other important processes tightly correlated with SGR, such as intra- and interspecific competition process, and substrates production and consumption process, which could effectively diminish the auto- and cross-correlation of stochastic processes of microbial populations, alleviating the intra- and inter-specific competitions. In artificial intelligence devices with LDUVR, these crucial succession processes can propel the microbial communities to generate and sustain a high species diversity. Finally, thorough *Monte Carlo* simulations were used to thoroughly confirm the idea. This research can build the theoretical groundwork, offer fresh viewpoints, and suggest potential microbial prevention strategies for the succession of microbial communities in LDUVR.

## 1. Introduction

Microbial diversity in the medical treatment environment, such as operating room, sickroom, treatment room, and injection , is often at a lower level, and all sections of the environment need to be properly cleaned, disinfected, and maintained. However, microbial diversity with high richness and evenness has been currently found in the artificial intelligence devices where periodic ultraviolet (UV) ray disinfection was used extensively, because various kinds of microbial species had been sampled and identified from the parts which were uneasily cleaned in the devices, such as screw, pulley, and backboard, where the microbial diversity is significantly higher than other parts of artificial intelligence devices. The microorganisms on the significant surface are killed by direct exposure to periodic high-dose UV radiation, nevertheless, those microorganisms colonized on the positions with a relatively long distance the from UV source can only receive periodic low-dose UV radiation (LDUVR) due to energy degradation [1, 2].

The indoor microorganisms are often combined with dust particles and exist in the form of aerosol suspending in the air and precipitating in artificial intelligence devices with periodic LDUVR [3]. The dust particles usually contain a small amount of macromolecular organic matters, which could be decomposed by the microbial community into monosaccharides, oligosaccharides, oligopeptides, amino acids, glycerol, fatty acids, and so on, which could be directly used as substrates for microbial growth and proliferation [4]. However, statistics show that the number of substrate types accessible for the microbial community in the medical treatment environment is about 10 at most, far less than the number of microbial species discovered in artificial intelligence systems with periodic LDUVR. Although only a few dominant species can coexist through substrate niche differentiation, the well-known competitive exclusion principle in ecology predicts that microbial species will compete fiercely over fewer varieties of substrates, making it impossible to create and maintain microbial diversity [5]. Although these phenomena were seen in artificial intelligence systems with periodic LDUVR, it is now unclear how the dynamic forces underpinning the microbial community succession work. The reason the microbiological variety can develop and persist in the artificial intelligence devices with periodic LDUVR is therefore still a mystery.

A negative disturbance for the microbial community succession in artificial intelligence devices could be the periodic LDUVR. The intermediate disturbance hypothesis has been put forth to suggest that species diversity will be higher in communities with moderate levels of perturbations than in communities with no perturbations or communities with rare or very frequent perturbations [6]. As is well known, ecosystem disturbance is defined as a relatively discrete event in time with frequency, intensity, and severity outside of a predictable range [7]. In a relatively simple environment with fluctuating temperature, for instance, many more species of phytoplankton have been observed to coexist, a phenomenon known as the “plankton paradox”. As an intermediate disturbance, fluctuating temperature may promote species diversity by reducing the pressure of dominant species on other species and allowing the latter to develop [8].

The periodic LDUVR can be viewed as an unfavorable factor with intermediate disturbance, causing microbial stochastic growth response (SGR) along with random variation of the crucial processes tightly correlated with SGR, such as intra- and inter-specific competition [8, 9]. This new dynamic mechanism is based on existing ecological investigations and drives microbial community succession with higher species diversity in artificial intelligence device with periodic LDUVR. In order to create and preserve high microbial diversity in artificial intelligence devices with periodic LDUVR, the periodic LDUVR may efficiently reduce the auto- and cross-correlation of stochastic processes of microbial populations.

In order to test the preceding hypothesis, in the research, the five most common genera, *Escherichia, Pseudomonas, Streptococcus, Staphylococcus*, *and Aeromonas* in artificial intelligence devices were periodically sampled and analyzed. To describe the dynamic mechanisms causing microbial community successions in artificial intelligence devices with periodic LDUVR, highly valid kinetic models expressed by differential equations with kinetic parameters obeying different normal distributions were established based on the proposed assumptions, experimental phenomena, and data [9]. Additionally, a large number of microbial species and substrates were computer-generated. By using a significant amount of *Monte Carlo* simulations along with experimental data, the hypothesis was properly validated and proven. The findings of this study could create the theoretical groundwork for understanding the ecological impact of LDUVR on the succession of microbial communities and offer a practical advice on microbial prevention and control in the presence of LDUVR.

## 2. Materials and Methods

### 2.1. Source of the Samples

The selected artificial intelligence devices were located in the medical treatment environment, which was clearly divided into two functional areas, UV disinfection room and controlled room, with good ventilation, and annual keeping temperature and humidity, respectively, at 19–24°C and 40%–50% through the central air-conditioning system.

As an experimental group, the microorganisms were sampled by cotton swabs from the screw, pulley, and backboard of the UV disinfection room in the artificial intelligence devices, the effective sampling area was 10 cm × 20 cm. A germicidal lamp (Ushio Inc. Tokyo, Japan) emitting primarily 254 nm ultraviolet radiation (UV) was routinely utilized for sterilization with the disinfection time from 8 am to 8 pm every day. The sampling place was 6.18 m away from the germicidal lamp, and exposed to periodic LDUVR. As a control group, the microorganisms were sampled from the same area without UV disinfection in the artificial intelligence devices, the effective sampling area was also 10 cm × 20 cm.

The sampling time is 1 day which is relatively a short period to capture transient dynamic characteristics of microbial abundances, and the last is 100 days. Ecologically, the dynamic processes of microbial populations in the artificial intelligence devices must be stochastic processes, since they are mainly dependent on intrinsic growth rates of microbial species, intra- and inter-specific competitions, and random environmental disturbances. Based on the stochastic process theory, if a long-time observation and record for microbial populations have been carried out, the accurate statistical characteristics of their stochastic processes, such as the mean, variance, auto- and cross-correlation function, and power spectral density (PSD), can be obtained from time-series data [10]. Therefore, 100 days are long enough for stochastic processes of microbial populations to go through all possible states. According to the classic Lotka–Volterra competition model, however, the dynamic characteristics of a species population are totally dependent on the intrinsic growth rate, and intra- and inter-specific competition; hence, the auto- and the cross-correlation function can fully reflect the intra- and inter-specific relationships and interactions, and disclose the dynamic mechanisms to drive microbial community succession in the artificial intelligence devices with periodic LDUVR. Therefore, only the auto- and the cross-correlation functions were calculated and used to analyze the stochastic process of microbial abundances [11, 12].

### 2.2. Analysis of Microbial Abundance and Diversity

The abundance of microbial samples was analyzed as the following steps:

1. Extracting microbial total DNA from the sample by using a powerful microbial DNA extraction kit (Power microbial® DNA Isolation Kit, MoBio)
2. High-throughput sequencing by means of an Illumina HiSeq platform using double-end sequencing
3. Performing quality control on preprocessed sequencing results using the DADA2 method
4. Dividing operational taxonomic units (OTUs) to assess the richness of the microbial community through the Chao1 Index
5. Annotating species for each sample and analyzing the composition of the microbial community abundance at the genus level
6. Calculating the microbial diversity based on the *Simpson index* and performing the overall *α* diversity analysis in conjunction with step (4)

The purified pooled sample was subjected to high-throughput sequencing analysis of bacterial rRNA genes utilizing the Illumina Hiseq 2500 platform (2250 paired ends) at Biomarker Technologies Corporation, Shanghai, China. These OTU sequences were classified taxonomically at various taxonomic levels using the RDP classifier and an 80 percent confidence criterion against the SILVA and UNITE databases.

### 2.3. Mathematical Modeling and Digital Simulations

Using the hypothesized theory, system dynamics, and experimental data, kinetic models of microbial community succession were created in this study [13]. Through digitally created *Monte Carlo* experiments, the microbial species and substrates were represented by model parameter vectors [14]. In order to simulate the scenario of microbial community succession in the controlled room and UV disinfection room with periodic LDUVR, respectively, the corresponding simulation models were established by MATLAB/Simulink based on these kinetic models. These stochastic parameters generated from the normal distribution would cause the stochastic processes of microbial populations to have different PSDs [15]. Digital simulations along with experimental data and phenomena were used to sufficiently validate and confirm the presented concept.

## 3. Results and Discussion

### 3.1. Dynamic Characteristics of Microbial Abundances

The microbial relative abundances of *Escherichia*, *Pseudomonas*, *Streptococcus*, *Staphylococcus* and *Aeromonas*, and the corresponding *Simpson Diversity Index* of the microbial community were analyzed and quantified (Figure 1), after periodical sampling from UV the disinfection room and controlled room of the artificial intelligence devices, respectively.

Based on stochastic processes of relative abundances of the five most common genera, calculate the autocorrelation function of the relative abundances stochastic process of each microbial genus sampled from the controlled room (Figure 2) and UV disinfection room (Figure 3), respectively.

Furthermore, the cross-correlation function between two microbial genus-relative abundance stochastic processes was also calculated and illustrated in Figures 4 and 5, respectively.

From Figures 1, 2, and 4, the auto- and cross-correlation function of microbial abundances stochastic processes as well as the *Simpson Index* of microbial community sampled from the controlled room are relatively large. Based on the classic *Lotka–Volterra* competition model and stochastic process theory, the auto- and cross-correlation function can indicate the influence of intra- and inter-specific competition strength on species population. The larger auto- and cross-correlation functions would indicate that intra- and inter-specific competition strongly correlated to dynamic characteristics of the species population [16]. Microbes would compete fiercely over a limited range of substrates through intra- and inter-specific competition; as a result, only a small number of species could coexist, and the majority of microbial species would go extinct due to competitive exclusion. Hence the *Simpson Index* also indicated low species diversity in the microbial community sampled from the controlled room (Figure 1).

From Figures 1, 3, and 5, however, the situation is exactly reversed, which suggested both the intra- and inter-specific competition were alleviated and the dynamic characteristics were fundamentally independent on the microbial intra- and inter-specific competition [17], and the *Simpson Index* also signified high species diversity in the microbial community sampled from the UV disinfection room.

### 3.2. Hypothesis of Microbial Diversity in Artificial Intelligence Devices with Periodic LDUVR

Even though experimental phenomena and data can be directly observed and measured, the underlying dynamic mechanisms created by relationships and interactions between microbial species and their biotic/abiotic environments cannot be directly identified and recognized; instead, they can only be understood by hypotheses that have been developed based on microbial ecology, experimental phenomena, and data, and sufficiently investigated by mathematical modeling and digital simulations [18].

The competitive exclusion scenario in the controlled room of the artificial intelligence device without LDUV could be imagined based on the following: microbial ecology, experimental data, and theoretical analyses. At the start of microbial community succession in the artificial intelligence devices, all populations grow exponentially. However, since substrate niches are regularly filled due to the quantity and kind of substrates being limited, their development rates must inevitably slow down. Due to inter-specific variations in intrinsic growth rates, competitive abilities, carrying capacities, and other factors, a turning point will manifest sooner or later. Some species will eventually stop developing while others will continue to do so, eventually excluding the former and driving it to extinction [19]. In order to understand the succession of the microbial population in UV disinfection, a new dynamic mechanism must be proposed. The following new hypothesis of dynamic mechanisms driving microbial community succession in artificial intelligence devices with periodic LDUVR was put forth to interpret new relationships and interactions between microbial species and their biotic/abiotic environments based on microbial ecology, easily observed experimental phenomena, and data.

As an adverse factor, the periodic LDUV could generate intermediate disturbance to cause stronger microbial SGR determining the microbial population size directly, and inevitably gives rise to stronger random variations of other processes, such as the intra- and inter-specific competition process and the substrates production and consumption process. The stronger stochastic fluctuation of microbial populations could effectively weaken the auto- and cross-correlation of stochastic processes of microbial populations, greatly alleviating intra- and inter-specific competition and increasing the possibility of a wide spectrum of the microbial species, according to the classic *Lotka–Volterra* competition model, which states that the intensity of microbial intra- and inter-specific competition only depends on the product of the species population size. As a result, a greater number of species can effectively cohabit under the intermediate disturbance induced by periodic LDUVR than that permitted under the competitive exclusion principle.

Instead, because of the relatively weak microbial populations' stochastic fluctuation caused by environmental background disturbances, which could lead to increased inter-specific competition and exclusion during microbial community succession in a controlled environment, the microbial diversity could not be formed or maintained at all.

### 3.3. Kinetic Model Derivation of Microbial Community Succession in Artificial Intelligence Device

The following rate equations were created to characterize the relationships and interactions between microbial species and their biotic/abiotic habitats in artificial intelligence devices based on the aforementioned premises and system dynamics.

#### 3.3.1. Rate Equations of Microbial Population Growth

Consider the scenario where *M* types of microbial species were colonized in the artificial intelligence device and *m* types of substrates were produced for direct utilization, satisfying *M* _*>*_ *m* to mimic the scenario where *M* types of microbial species were much more numerous than *m* types of substrates in the artificial intelligence devices. The *i-th* microbial population (*x*_*i*_) and the *k-*th substrate amount (*S*_*k*_) produced by microbial breakdown were thus the state variables in the kinetic model. The *i-th* microbial population growth rate (*v*_*bi*_) was formulated by Monod equations as follows:

(1) $$\begin{array}{c} v_{bi}=\left[\mu_{i}+\varepsilon_{1}\left(t\right)\right]x_{i}\left(t\right)\sum_{k=1}^{m}\frac{S_{k}\left(t\right)}{K_{ik}+S_{k}\left(t\right)}, \end{array}$$

where *K*_*ik*_ is the half-saturation constant of the *i-th* microbial population growth on the *k-th* substrate, *μ*_*i*_ is the specific growth rate of the *i-th* microbial population, *ε*_1_(*t*) is normally distributed random numbers, and *μ*_*i*_ represents the environmental disturbance .

#### 3.3.2. Rate Equations of Microbial Intra- and Inter-specific Competition

The traditional *Lotka–Volterra* competition model was used to develop the rate equations for intraspecific and inter-specific competition. The rates of intraspecific competition within the *i-th* microbial species (*v*_*ai*_) were expressed as follows:

(2) $$\begin{array}{c} v_{ai}=\left[\alpha_{i}+\varepsilon_{2}\left(t\right)\right]x_{i}^{2}, \end{array}$$

where *α*_*i*_ is the intraspecific competition inhibition coefficient of the *i-th* microbial species and *ε*_2_(*t*) is a set of randomly generated values with normal distribution and is a proxy for *α*_*i*_ environmental disturbance.

The following could be stated as the rates of inter-specific competition between the *i-th* and *j-th* microbial species (*v*_*ei*_):

(3) $$\begin{array}{c} v_{ei}=\sum_{i\neq j}^{M}\left[\beta_{ij}+\varepsilon_{3}\left(t\right)\right]x_{i}\left(t\right)x_{j}\left(t\right), \end{array}$$

where *β*_*ij*_ stands for the inter-specific competition inhibition coefficient of the *j-th* microbial population on the growth rate of the *i-th* microbial population and *ε*_3_(*t*) is a random number with a normal distribution and reflects *β*_*ij*_ environment.

#### 3.3.3. Metabolism Rate of Microbial Population

The following could be used to express the metabolic rate of the *i-th* microbial population (*v*_*di*_):

(4) $$\begin{array}{c} v_{di}=d_{i}x_{i}, \end{array}$$

where *d*_*i*_ is the metabolism coefficient of the *i-th* microbial population.

#### 3.3.4. Substrates Production and Consumption Rate

Furthermore, the production rate of the *k-th* substrate by the *i-th* microbial species through microbial decomposition (*v*_*pki*_) could be specified as follows [20]:

(5) $$\begin{array}{c} v_{pki}=r_{k}\sum_{i=1}^{M}\left[c_{i}+\varepsilon_{4}\left(t\right)\right]\frac{x_{i}}{Z_{i}+x_{i}}, \end{array}$$

where *r*_*k*_ is the proportion of the *k-th* substrate to the total substrates produced by microbial decomposition, *c*_*i*_ is the maximum rate of substrate production of the *i-th* microbial species with the half-saturation constant *Z*_*i*_, and *ε*_4_(*t*) is normally distributed random numbers and represents the environmental disturbance to *c*_*i*_.

Similarly, the consumption rate of the *k-*th substrate during the *i-th* microbial population growth (*v*_*cki*_) could be specified as follows:

(6) $$\begin{array}{c} v_{cki}=h_{k}\sum_{i=1}^{M}\left[\gamma_{i}+\varepsilon_{5}\left(t\right)\right]v_{bi}, \end{array}$$

where *h*_*k*_ is the ratio of the *k-th* substrate to the total number of substrates consumed by the microbial community, *γ*_*i*_ is the substrates consumption coefficient of the *i-th* microbial population, *ε*_5_(*t*) is normally distributed random numbers, and *γ*_*i*_ represents the environmental disturbance.

#### 3.3.5. General Kinetic Model Obtained from Rate Equations

A top-down state-space model with *M* + *m* first-order nonlinear ODEs of microbial community succession in the artificial intelligence devices was built based on the prior analysis and establishing rate equations [21].

The first-order kinetic equation of the *i-th* microbial population can be stated as follows, with reference to (1)–(4):

(7) $$\begin{array}{c} \frac{\text{d}x_{i}\left(t\right)}{\text{d}t}=v_{bi}-v_{ai}-v_{ei}-v_{di}\\ =\left[\mu_{i}+\varepsilon_{1}\left(t\right)\right]x_{i}\left(t\right)\sum_{k=1}^{m}\frac{S_{k}\left(t\right)}{K_{ik}+S_{k}\left(t\right)}-\left[\alpha_{i}+\varepsilon_{2}\left(t\right)\right]x_{i}^{2}-\sum_{i\neq j}^{M}\left[\beta_{ij}+\varepsilon_{3}\left(t\right)\right]x_{i}\left(t\right)x_{j}\left(t\right)-d_{i}x_{i}. \end{array}$$

The first-order kinetic equation of the *k-th* substrate can be expressed as follows with reference to (1), (5), and (6):

(8) $$\begin{array}{c} \frac{\text{d}S_{k}\left(t\right)}{\text{d}t}=v_{pki}-v_{cki}=r_{k}\sum_{i=1}^{M}\left[c_{i}+\varepsilon_{4}\left(t\right)\right]\frac{x_{i}}{Z_{i}+x_{i}}-h_{k}\sum_{i=1}^{M}\left[\gamma_{i}+\varepsilon_{5}\left(t\right)\right]\left[\mu_{i}+\varepsilon_{1}\left(t\right)\right]x_{i}\left(t\right)\sum_{k=1}^{m}\frac{S_{k}\left(t\right)}{K_{ik}+S_{k}\left(t\right)}. \end{array}$$

### 3.4. Microbial Species and Substrates Computer-Generated for Simulation

The *i-th* microbial species could be represented by a parameter vector (*μ*_*i*_, *α*_*i*_, *β*_*ij*_, *K*_*ik*_, *d*_*i*_, *c*_*i*_, *γ*_*i*_, *Z*_*i*_), and the *k-th* substrate could be denoted by a parameter vector (*r*_*k*_, *h*_*k*_), as the parameters in kinetic models (equations (7) and (8)) of microbial community succession can embody specific biological and ecological characteristics tightly dependent on specific microbial genomes. These parameters could be acquired using parameter estimation uniformly and independently by random selection from defined parametric intervals [22] (Table 1).

In this study, the 5∼15 different types of substrates and 20∼50 different microbial species were produced stochastically by computers and inserted into kinetic models (equations (7) and (8)). This method allowed for the formulation of kinetic models with various dimensions for theoretical investigation of the succession of microbial communities in artificial intelligence devices and the validation of the hypothesis regarding the emergence and preservation of microbial diversity as a result of intermediate disturbance brought on by periodic LDUVR.

A large scale of *Monte Carlo* simulations was then carried out to confirm the proposed hypothesis on the formation and maintenance of microbial biodiversity in the artificial intelligence device with periodic LDUVR. Before digital simulation, simulation methods and other options were properly set [21], according to the complexity of kinetic models, accuracy, convergence speed, and computational cost.

### 3.5. *Monte Carlo* Simulations for Microbial Community Successions

The simulation model was correspondingly established on the Matlab/Simulink platform to conduct *Monte Carlo* simulations to support the proposed hypothesis on microbial community succession in artificial intelligence devices based on kinetic models (equation (7) and (8)) of microbial community succession in artificial intelligence devices (Figure 6) [23].

Figure 6 shows how the random number blocks were used to simulate environmental disturbances whose PSD was applied for assessments of the strength of disturbances. The PSD was set at reasonably mild values generated at random from the value range. The simulation results fully demonstrated that the number of coexisting microbial species was far greater than the types of substrates produced by microbial decomposition, and the microbial populations generate almost independent stochastic processes via desultorily transient responses (Figure 7). These dynamic behaviors could significantly reduce intra- and inter-specific competition [24, 25]. It will be advantageous for a large number of microbial species to dwell in artificial intelligence devices with periodic LDUVR to concurrently boost the richness and evenness of the microbial community.

It is important to note that the digital simulation results of the microbial community succession patterns that emerged in the artificial intelligence device with periodic LDUVR, as shown in Figure 7, are quite universal and general since these simulation results only depend on the structure of kinetic models, specifically the interactions and relationships between microbial populations and their biotic/abiotic environments in the artificial intelligence devices with periodic LDUVR.

Due to the PSD's modest setting, however, values chosen at random from the value range of the simulation results suggested that, subjected to competitive exclusion, the majority of microbial species would eventually go extinct, with only a few species whose number is no more than the substrate types produced by microbial decomposition being able to coexist (Figure 8), due to drastic intra- and inter-specific competition reflected in strong auto- and cross-correlation of stochastic without LDUVR to simulate the scenarios with weak disturbance caused by environmental background disturbances.

## 4. Conclusions

We theoretically provide a hypothesis on the production and preservation of microbial diversity in the artificial intelligence devices with intermediate disturbance brought on by periodic LDUVR based on microbial ecology, experimental phenomena, and data. The periodic LDUVR could produce intermediate disturbance that would lead to stronger microbial SGR along with stronger random process variations of substrate production and consumption. This would significantly reduce the auto- and cross-correlation of microbial populations stochastic processes and effectively alleviate intra- and inter-specific competition to form and maintain a microbial community with higher richness. The hypothesized hypothesis was then quantified using a collection of kinetic models written by differential equations with parameters obeying various normal distributions. Finally, a significant number of *Monte Carlo* simulations were performed to sufficiently validate and confirm the proposed theory. The findings of this study could create the theoretical groundwork for understanding the ecological impact of LDUV on the succession of microbial communities and offer practical advice on microbial prevention and control in the context of LDUVR.

## Figures and Tables

**Figure 1:** Stochastic processes of 5 genera abundances and the *Simpson Index* of microbial community respectively sampled from the controlled room and UV disinfection room.

**Figure 2:** Autocorrelation function of the relative abundances stochastic process of each microbial genus sampled from the controlled room.

**Figure 3:** Autocorrelation function of the relative abundances stochastic process of each microbial genus sampled from UV disinfection room.

**Figure 4:** Cross-correlation function between two microbial genus-relative abundance stochastic processes from the controlled room.

**Figure 5:** Cross-correlation function between two microbial genus-relative abundance stochastic processes from the UV disinfection room.

**Figure 6:** Part of the simulation model of microbial community succession in artificial intelligence devices.

**Figure 7:** Microbial community succession pattern in artificial intelligence devices with periodic LDUVR.

**Figure 8:** Microbial community succession pattern in artificial intelligence devicess without LDUVR.

**Table 1:** Parametric intervals in the kinetic models.

Parameter	Unit	Parametric interval		Significance
		Without LDUVR	With LDUVR	
*μ*_*i*_	h^−1^	(0.24, 1.36)		The *i-th* microbial species' particular growth rate.
*α*_*i*_	(log_10_ CFU^−1^) ml·h^−1^	(0.05, 1)		The *i-th* microbial species' intraspecific competition coefficient.
*β*_*ij*_	(log_10_ CFU^−1^) ml·h^−1^	(0.16, 1)		The *j-th* microbial species' inter-specific competition coefficient on the *i-th* microbial species' growth rate.
*c*_*i*_	mg·h^−1^	(136.23, 518.76)		The *i-th* microbial species' highest rate of substrate production
*γ*_*i*_	mg (log_10_ CFU)^−1^ ml	(3.32, 12.55)		The consumption coefficient of substrates by the *i-th* microbial species
*ε*_*1*_	W·Hz^−1^	(0, 2)	[2, 10]	Environmental disturbance to *μ*_*i*_
*ε*_*2*_	W·Hz^−1^	(0, 2)	[2, 10]	Environmental disturbance to *α*_*i*_
*ε*_*3*_	W·Hz^−1^	(0, 2)	[2, 10]	Environmental disturbance to *β*_*ij*_
*ε*_*4*_	W·Hz^−1^	(0, 2)	[2, 10]	Environmental disturbance to *c*_*i*_
*ε*_*5*_	W·Hz^−1^	(0, 2)	[2, 10]	Environmental disturbance to *γ*_*i*_
*K*_*ik*_	mg	(1.23·10^5^, 1.82·10^5^)		The *i-th* microbial species' half-saturation constant while growing on the *k-th* substrate.
*d*_*i*_	h^−1^	(0.03, 0.58)		The *i-th* microbial species' metabolic coefficient.
*Z*_*i*_	(log_10_ CFU) ml^−1^	(42, 177)		The substrates produced by the *i-th* microbial species' half-saturation constant.
*r*_*k*_	%	(0, 80)		The percentage of all substrates generated by the microbial population to the *k-th* substrate.
*h*_*k*_	%	(0, 80)		The proportion of the *k-th* substrate to total substrates consumed by microbial community.

## Data Availability

The data used to support the findings of this study are available from the corresponding author upon request.
